The article "Piper betle induces phase I & II genes through Nrf2/ARE signaling pathway in mouse embryonic fibroblasts derived from wild type and Nrf2 knockout cells" was published in 2014. Journal: BMC Complement Altern Med.

# *Piper betle* induces phase I & II genes through Nrf2/ARE signaling pathway in mouse embryonic fibroblasts derived from wild type and Nrf2 knockout cells

**DOI:** 10.1186/1472-6882-14-72

**Published:** 2014-02-23

**Authors:** Wan Nuraini Wan Hasan, Mi-Kyoung Kwak, Suzana Makpol, Wan Zurinah Wan Ngah, Yasmin Anum Mohd Yusof

**Affiliations:** 1 Department of Biochemistry, Faculty of Medicine, Universiti Kebangsaan Malaysia, Jalan Raja Muda Abdul Aziz, 50300 Kuala Lumpur, Malaysia; 2 College of Pharmacy, The Catholic University of Korea, Bucheon, Gyeonggi-do 420-743, Korea

**Keywords:** Nrf2, PB, ARE, NQO1, HO-1, GST. SOD1

## Abstract

**Background:**

Nuclear factor-erythroid 2 p45 related factor 2 (Nrf2) is a primary transcription factor, protecting cells from oxidative stress by regulating a number of antioxidants and phase II detoxifying enzymes. Dietary components such as sulforaphane in broccoli and quercetin in onions have been shown to be inducers of Nrf2. *Piper betle* (PB) grows well in tropical climate and the leaves are used in a number of traditional remedies for the treatment of stomach ailments and infections among Asians. The aim of this study was to elucidate the effect of *Piper betle* (PB) leaves extract in Nrf2 signaling pathway by using 2 types of cells; mouse embryonic fibroblasts (MEFs) derived from wild-type (WT) and Nrf2 knockout (N0) mice.

**Methods:**

WT and N0 cells were treated with 5 and 10 μg/ml of PB for 10 and 12-h for the determination of nuclear translocation of Nrf2 protein. Luciferase reporter gene activity was performed to evaluate the antioxidant response element (ARE)-induction by PB. Real-time PCR and Western blot were conducted on both WT and N0 cells after PB treatment for the determination of antioxidant enzymes [superoxide dismutase (SOD1) and heme-oxygenase (HO-1)], phase I oxidoreductase enzymes [NAD(P)H: quinone oxidoreductase (NQO1)] and phase II detoxifying enzyme [glutathione S-transferase (GST)].

**Results:**

Nuclear translocation of Nrf2 by PB in WT cells was better after 10 h incubation compared to 12 h. Real time PCR and Western blot analysis showed increased expressions of Nrf2, NQO1 and GSTA1 genes with corresponding increases in glutathione, NQO1 and HO-1 proteins in WT cells. Reporter gene ARE was stimulated by PB as shown by ARE/luciferase assay. Interestingly, PB induced SOD1 gene and protein expressions in N0 cells but not in WT cells.

**Conclusion:**

The results of this study confirmed that PB activated Nrf2-ARE signaling pathway which subsequently induced some phase I oxidoreductase, phase II detoxifying and antioxidant genes expression via ARE reporter gene involved in the Nrf2 pathway with the exception of SOD1 which may not be dependent on this pathway.

The article "Piper betle induces phase I & II genes through Nrf2/ARE signaling pathway in mouse embryonic fibroblasts derived from wild type and Nrf2 knockout cells" was published in 2014. Journal: BMC Complement Altern Med.

## Background

*Piper betle* L. (PB) from Piperaceae family grows well in South East Asia. The leaves of PB are used as masticatory in many Asian countries including Malaysia. Eugenol and hydroxychavicol are two bioactive compounds in PB that have been reported to have antioxidant and anti-inflammatory properties [1,2]. The highest phytochemical present in water extract of PB leaves is hydroxychavicol which contributed to its antioxidant activity [2]. PB improved antioxidant status by increasing activities of free radical–detoxifying enzymes such as superoxide dismutase, catalase, and glutathione peroxidase during aging in erythrocyte of C57BL/6 mice [3] and increased the levels of nonenzymatic antioxidants such as reduced glutathione in liver and kidney of ethanol-treated rats [4]. Aqueous extract of PB leaves improved antioxidant potential by increasing SOD and catalase activity and also reducing lipid peroxidation in liver and kidney of diabetic-induced Wistar rats [5]. A recent finding showed that PB inhibited proliferation of breast cancer cell lines, MCF-7 and increased antioxidant activities such as SOD1 and CAT [6].

Oxidative stress results from an imbalance between excess production of ROS and limited cellular antioxidant defense [7]. The basic leucine-zipper transcription factor nuclear factor-erythroid 2 p45-related factor 2 (Nrf2) plays a vital role in protecting cells from oxidative stress [8,9]. Nrf2 is normally sequestered in the cytoplasm as an inactive complex by interaction with its repressor Keap1 [10]. There are two prevailing models which proposed how Nrf2 is released from Keap1 in response to oxidative stress; (1) the ‘hinge and latch’ model, in which Keap1 modifications in thiol residues of Keap1 disrupt the interaction with Nrf2 causing misalignment of the lysine residues within Nrf2 that can no longer be polyubiquitinylated, and (2) the model in which thiol modification causes dissociation of Cul3 from Keap1 [11]. In both models, the inducer-modified and Nrf2-bound Keap1 is inactivated and, consequently, newly synthesized Nrf2 proteins bypass Keap1 and translocate into nucleus, bind to the Antioxidant Response Element (ARE) and leads to transcriptional induction of Nrf2 target genes such as heme oxygenase-1 (HO-1), superoxide dismutase (SOD1), catalase (CAT), NAD(P)H quinone oxidoreductase (NQO1), glutathione S-transferase (GST), and including glutathione biosynthesis enzymes glutathione cysteine ligase modifier subunit (GCLM) and glutathione cysteine ligase catalytic subunit (GCLC) [11-18].

Some phytochemical compounds that have been reported to activate the Nrf2/ARE pathway include sulforaphane from broccoli [19,20], quercetin from onions [21] and epigallocatechin-3-gallate from green tea [20]. To our knowledge no information is available on the association of PB with the Nrf2/ARE signalling pathway. The aim of this experiment was to evaluate whether PB can modulate Nrf2/ARE pathway with subsequent increase in phase 2 and endogenous antioxidant enzymes using mouse embryonic fibroblast (MEF) from wild-type and Nrf2 knockout mice.

The article "Piper betle induces phase I & II genes through Nrf2/ARE signaling pathway in mouse embryonic fibroblasts derived from wild type and Nrf2 knockout cells" was published in 2014. Journal: BMC Complement Altern Med.

## Methods

### Materials

Mouse embryonic fibroblasts (MEFs) were a kind gift from Kwak Mi-kyoung (The Catholic University of Korea, Bucheon, South Korea) and Nobunao Wakabayashi (University of Pittsburgh, USA).who have prepared the cell line from wild type (Nrf2^+/+^) and *nrf2*-disrupted (Nrf2^-/-^) ICR mice [22]. Reporter plasmid containing NQO1 ARE-luciferase [23] was also a kind gift from Kwak Mi-kyoung.

### Cell culture

MEFs cells were cultured in Iscove’s modified Dulbecco’s medium (Invitrogen, USA) supplemented with 10% FBS (PAA, USA), 10 unit/ml penicillin-streptomycin and 2.5 μg amphoterecin-B (PAA, USA).

### MTS assay

Cells were plated at a density of 5 × 10^3^ cells/well in 96-well plates. After 24 h of incubation the cells were treated with various concentrations of aqueous PB extract. Then, 20 μl MTS solution (Promega, USA) was added to each well and the cells were further incubated for 4 h. The absorbance was measured at 490 nm using a Versamax microplate reader (Sunnyvale, CA, USA).

### Aqueous extraction of *Piper betle* leaves

Dried PB leaves were purchased from Ethno Resources Company (Sungai Buloh, Selangor, Malaysia) and confirmation of identification of the plant was obtained from Herbarium, Universiti Kebangsaan Malaysia, Bangi with voucher number UKMB 29768. Aqueous extraction of PB was prepared according to Pin et al. [2] with some modifications. Briefly, the leaves were ground into powder and concentration of 10% PB was prepared and the extraction process was done using a Soxhlet Extractor (Eyela, Japan). The PB aqueous extract was freeze dried (Labconco, USA). into powder form and stored at 4°C until further use.

### Reporter plasmid transfection and luciferase activity measurement

Cells were transfected with plasmids at 50% confluence using Welfect-Ex Plus transfection reagent (WelGene, Daegu, South Korea). Briefly, cells were incubated with the transfection complex containing 0.5 μg ARE-luciferase plasmid, 0.05 μg pRLtk control plasmid, and the transfection reagent (2 μg Welfect-Ex and 1.5 μg Enhancer-Q) in serum-and antibiotic-free OptiMEM (Invitrogen, USA). Transfection was continued for 18 h; the cells were then recovered in complete medium for the next 8 h. The cells were treated with 5 and 10 μg/ml of PB for 24 h and were then lysed with lysis buffer [RIPA buffer (Sigma, USA) and protease inhibitor cocktail tablet (Roche, Switzerland)]. Luciferase activities from firefly and Renilla luciferases in total cell lysates were determined using a Dual-Luciferase Assay kit (Promega, Wisconsin, USA) with a 20/20n luminometer (Turner Biosystems, Sunnyvale, CA, USA). Wild-type cells were treated with 5 μM sulforaphane (SFN) for 6 h as a positive control.

The article "Piper betle induces phase I & II genes through Nrf2/ARE signaling pathway in mouse embryonic fibroblasts derived from wild type and Nrf2 knockout cells" was published in 2014. Journal: BMC Complement Altern Med.

### Preparation of nuclear extracts

For Nrf2 detection in the nucleus, cells were grown with a density of 6×10^5^ and were treated with 5 and 10 μg/ml of PB for 10 and 12 h. After treatment, the cells were washed with cold-PBS. Crude nuclear fractions were obtained by lysing cells in homogenization buffer [2 M sucrose, 1 M Hepes, 2 M MgCl_2_, 2 M KCl, 30% glycerol, 0.5 M EDTA, 1 M dithiothreitol, protease inhibitor cocktail (Sigma, USA), and 0.2% NP-40 (Sigma, USA)], scraped off, vortexed for 30 min at 4°C and followed by centrifugation at 12,000 × g for 15 min. Protein concentration was determined using Bio-Rad protein assay dye (Hercules, CA).

### RNA extraction and quantitative real-time PCR

Cells were seeded in 6-well plates at 2x10^5^/well and cultured for 24-h. After 24-h treatment with 5 and 10 μg/ml of PB extract, the cells were washed with PBS and RNA was isolated using TRI reagent (Molecular Research Centre, Inc., USA). PCR amplification was performed with a thermal cycler (BioRad, USA). The mRNA level was quantified by Bio-Rad iCycler and the condition for PCR amplification was 40 cycles of 10 sec at 95°C for denaturation and 30 sec at 56°C for annealing. The primers sequences for the genes are listed in Table 1 and were synthesized by FirstBase (Singapore).

**Table 1:** Oligonucleotide sequences for real-time PCR of murine phase 2 and antioxidative enzymes

**Gene**		**Sequences (5’-3’)**	**Accession No**
β-actin	Forward	GAAGAGCTATGAGCTGCCTGA	NM_007393.3
	Reverse	GCACTGTGTTGGCATAGAGGT	
Nrf2	Forward	GAACTGTAGGAAAAGGAAGC	U20532
	Reverse	GAGTATTCACTGGGAGAGTA	
NQO1	Forward	TTCTCTGGCCGATTCAGAGT	X13356
	Reverse	GGCTGCTTGGAGCAAAATAG	
SOD1	Forward	CGGATGAAGAGAGGCATGTT	Z18857
	Reverse	CACCTTTGCCCAAGTCATCT	
GSTA1	Forward	CCGTTACTTGCCTGCCTTTG	NM_145740
	Reverse	CTTCTTCACATTGGGGAGGCT	

### Western blot analysis

Cells were incubated with 5 and 10 μg/ml of PB for 24 h for detection of NQO1, HO-1 and SOD1 protein expression. Briefly, 2×10^4^ of cells were cultured in 60 mm petri dish and after 24 h treatment, the cells were lysed by using lysis buffer [RIPA buffer (Sigma, USA) and protease inhibitor cocktail tablet (Roche, Switzerland)] to extract the protein from cytosol. Finally, the cell lysates were centrifuged at 16,100 × g for 30 min and supernatant was stored at -80°C. Both cell lysates from cytosolic and nuclear extract were loaded on 12 or 15% SDS–polyacrylamide gels and separated by electrophoresis at 70 V using Mini-PROTEAN 3 cell system (BioRad, USA). Proteins on gels were transferred to PVDF membranes (Amersham Biosciences, UK) and the membranes were blocked with 5% skim milk in TPBS buffer (8 g/L NaCl, 0.2 g/L KCl, 1.44 g/L Na_2_HPO_4_, 0.24 g/L KH_2_PO_4_, and 2 ml/L Tween 20) for 1 h. Antibodies against β-actin, lamin B, SOD1 and NQO1 were purchased from Santa Cruz Biotechnology (Santa Cruz, CA, USA) while antibodies against HO-1 and HO-1 were purchased from Abcam, (Cambridge, UK). Primary antibody incubation was performed overnight followed by incubation with secondary antibody conjugated to horseradish peroxidase (SantaCruz, USA) for 1 h. Detection of proteins was performed using the Enhanced Chemiluminescence reagent (Amersham Biosciences, UK).

The article "Piper betle induces phase I & II genes through Nrf2/ARE signaling pathway in mouse embryonic fibroblasts derived from wild type and Nrf2 knockout cells" was published in 2014. Journal: BMC Complement Altern Med.

### Statistical analysis

Statistical analysis was conducted using the SPSS software for Windows, version 16.0. Differences between mean values of multiple groups were analyzed by one-way analysis of variance (ANOVA) with Tukey’s HSD post-hoc test. Confidence level at the 95% (*P* < 0.05) was considered statistically significant.

## Results

### Viability of WT and N0 cells to PB treatment

MTS assay was performed to measure cell viability after 24 h treatment with increasing doses of PB. N0 cells displayed almost 2-fold increased sensitivity (IC_50_) to PB compared to WT cells (Figure 1). This result indicated that N0 cells are more susceptible to cytotoxicity of PB treatment compared to WT cells.

**Figure 1:** **N0 cells display increased toxicity to PB aqueous extract.** WT and N0 cells were treated with increasing doses of PB for 24 h and cell viability was assessed by the MTS assay. Mean cell viability are expressed as percentage of control. Data represent ± S.E.M from three independent experiments. ^a^*P* < 0.05, compared to control; ^b^*P* < 0.05, compared to WT cells at the same concentration.

### Translocation of Nrf2 to nucleus by PB

To verify dissociation of Nrf2 from Keap1, we measured the translocation of Nrf2 protein into the nucleus in both WT and N0 cells after 10 and 12 h treatment with PB. After 10 h of 10 μg/ml PB treatment, nuclear Nrf2 level in WT cells was significantly different (p < 0.05) compared to N0 cells while treatment for 12 h resulted in no significant changes of Nrf2 proteins between the two types of cells (Figure 2). When compared to with the positive control of 5 μM sulforaphane on WT for 6 h, PB treatment for 10 h activated Nrf2 and translocated it into the nucleus at a lower level compared to SFN. This suggested that PB activated Nrf2 protein which subsequently translocated from the cytosol to the nucleus better after 10 h treatment when compared to 12 h treatment.

The article "Piper betle induces phase I & II genes through Nrf2/ARE signaling pathway in mouse embryonic fibroblasts derived from wild type and Nrf2 knockout cells" was published in 2014. Journal: BMC Complement Altern Med.

**Figure 2:** **Western blot analysis of nuclear translocation of Nrf2 by PB in Mouse Embryonic Fibroblast (MEF) of wild type (WT) and Nrf2 knockout cells (N0) for 10 and 12 h treatment.** The blots shown are examples of three separate experiments **(A)** of Nrf2 protein in the nucleus after 10 and 12 h. SFN treatment for 6 h serve as the positive control for Nrf2 activation and translocation into the nucleus. MEF cells were treated with PB (5 and 10 μg/ml) for **(B)** 10 h **(C)** 12 h, after which the cells were gathered and Nrf2 protein was extracted from the nucleus. Lamin B was used as internal control. Data represent ± S.E.M from three independent experiments. ^a^*P* < 0.05, compared to control WT cells; ^b^*P* < 0.05, compared to respective WT cells group.

### ARE-luciferase reporter gene activity

The inducer effect of PB on antioxidant and phase 2 genes mediated via ARE was verified as shown in Figure 3. Both WT and N0 cells were transfected with luciferase reporter plasmid containing the *NQO1*-ARE. Treatment of WT cells transfected with *NQO1*-ARE at 10 μg/ml of PB for 24-h showed 1.6-fold increase in luciferase activity compared to control (Figure 3).

**Figure 3:** **ARE-driven luciferase activities after treatment with PB in MEFs WT and N0 cells.** The cells were transfected with the luciferase reporter plasmid containing the NQO1 ARE and were treated with PB (5 and 10 μg/ml) or SFN (5 μM) for 24 h. Measurement of luciferase activities was performed using the Dual luciferase activities and Firefly luciferase levels were normalized to Renilla luciferase levels. Data represent ± S.E.M from four independent experiments. ^a^*P* < 0.05, compared to control WT cells; ^b^*P* < 0.05, compared to respective WT cells group.

### Effects of PB on gene expressions of antioxidants, phase I and phase II detoxifying enzymes

To explore the effect of PB on Nrf2-genes, WT and N0 cells were treated with PB and transcript levels for Nrf2, NQO1, SOD and GSTA1 genes were assayed via real time PCR. At the baseline, Nrf2, NQO1 and GSTA1 genes were highly expressed in WT cells compared to N0 cells (Figure 4). Treatment with PB at 10 μg/ml for 24-h for both type of cells significantly increased Nrf2, NQO1 and GSTA1 genes expression in WT, but not in N0 cells. SOD1 gene expression was significantly greater in N0 cells compared to WT cells at the baseline. However, when the cells were treated with PB, there was no significant difference in SOD1 expression between WT and N0 cells.

The article "Piper betle induces phase I & II genes through Nrf2/ARE signaling pathway in mouse embryonic fibroblasts derived from wild type and Nrf2 knockout cells" was published in 2014. Journal: BMC Complement Altern Med.

**Figure 4:** **Transcript levels for Nrf2, NQO1 and SOD1 genes following 5 and 10 μg/ml of PB treatment for 24-h.** RNAs were isolated and reverse transcribed to cDNA, then amplified by real-time PCR detection system to measure mRNA levels for beta actin, Nrf2 **(A)**, NQO1 **(B)** and SOD1 **(C)**, HO-1 **(D)** and GSTA1 **(E)**. Target genes were normalized to beta actin. Data represent ± S.E.M from three independent experiments. ^a^*P* < 0.05, compared to control WT cells; ^b^*P* < 0.05, compared to respective WT cells group.

### Effects of PB on NQO1 and HO1 protein expressions

To verify the induction of PB on Nrf2-regulated proteins, we measured the expression of NQO1 and HO-1 proteins by Western blot technique. At the basal level, NQO1 and HO-1 proteins were significantly expressed in WT cells compared to N0 cells (Figure 5A). When the cells were treated with 10 μg/ml PB for 24-h, NQO1 and HO-1 proteins were significantly increased in WT cells, but not in N0 cells. SOD1 protein however, was significantly expressed in N0 cells (Figure 5D) in accordance with the expression of SOD1 genes (Figure 4C) with PB treatment. However there was no significant difference in SOD1 expression between WT and N0 cells.

**Figure 5:** **Western blot of NQO1, HO-1 and SOD1 proteins in WT and N0 cells treated with PB (5 and 10 μg/ml).** The blots shown are examples of three separate experiments **(A)** from 20 μg cytosolic proteins and relative intensities over β-actin for NQO1 **(B)**, HO-1 **(C)** and SOD1 **(D)** protein expression after 24 h treatment of PB. SFN treatment at 5 μM was used as positive control. Data represent ± S.E.M from three independent experiments. ^a^*P* < 0.05, compared to control WT cells; ^b^*P* < 0.05, compared to respective WT cells group.

## Discussion

The underlying mechanism by which local plant *Piper betle* (PB) stimulates Nrf2 pathway has yet not been elucidated. Our results on NQO1-ARE luciferase activity, mRNA, phase I oxidoreductase and phase II detoxifying enzymes showed that PB induced Nrf2/ARE pathway.

This study illustrated that Nrf2 deficiency in MEF cells (N0) resulted in increased cytotoxicity with PB treatment compared to WT cells. Hydroxychavicol which is found in PB was shown to exert antioxidant activity at low concentration but display pro-oxidant effect at concentration higher than 0.1 mM [24]. Similarly, Nrf2^-/-^ MEF cells were shown to be more sensitive to SFN treatment, peroxides, anti-cancer drugs (Displatin) and compounds that generate free radical compared to Nrf2^+/+^ MEF cells [25].

The Nrf2-Keap1-ARE signaling system is central to the induction of phase 2 genes by electrophiles and antioxidants [16,17,20,21]. We showed that PB was able to activate Nrf2 and translocated into the nucleus, with increased expression of NQO1 and HO-1 genes and proteins. We postulate that the mechanism of interaction between PB and Nrf2-Keap1 complex may mimic the action of other Nrf2 inducers such as sulforaphane and *Gingko biloba* extract. Keap1 protein contains multiple cysteine residues and specifically C257, C273, C297 and C288 were shown to be the most reactive residues that can interact with phase 2 inducers including sulforaphane [10]. Upon exposure to inducers, the reactive cysteine residues form intermolecular disulfide bonds and change its conformation which leads to dissociation of Nrf2 from Keap1, translocating Nrf2 into the nucleus, and activating the expression of phase 2 genes [26]. *Ginkgo biloba* extract stimulated Nrf2, and translocated it into the nucleus with subsequent increase in phase 2 genes such as GCLC, GST and NQO1 through Keap1-Nrf2-ARE signaling pathway in Hepa1c1c7 and HepG2 cells [27]. The active compound in coffee, 5-*O*-caffeoylquinic acid (CGA) modulates Nrf2 nuclear translocation and ARE-dependent gene expression such as HO-1, Nrf2, GST, γGCL in HT29 cells [28].

The article "Piper betle induces phase I & II genes through Nrf2/ARE signaling pathway in mouse embryonic fibroblasts derived from wild type and Nrf2 knockout cells" was published in 2014. Journal: BMC Complement Altern Med.

In this study, we showed that Nrf2 translocation is better at 10 h incubation of PB, and for ARE induction, genes and proteins expression, we incubated the cells with PB for 24 h, which is similar to other studies [27,29]. Sulforaphane caused nuclear translocation of Nrf2 after 6 h treatment by Western blotting; however immunocytochemistry data revealed that translocation of Nrf2 in the nucleus was not seen in many cells at 6 h treatment compared to 24 h incubation that displayed high amount of Nrf2 in the nucleus of human keratinocytes cells [29].

The antioxidant response elements (ARE) are a cis-acting enhancer sequence located in the 5’-flaking promoter region of antioxidant and detoxifying genes such as GST, HO-1, GCLC and NQO1 [30-35]. The luciferase reporter assay further confirmed that PB induced ARE promoter region in the nucleus. Our results are supported by Shin et al. [16] who reported that sulforaphane, a well known Nrf2 activator, increased luciferase activity 3.5-fold in rat kidney epithelial NRK cells. Other dietary agents which activate ARE reporter gene with increased expression of Nrf2-targeted genes such as NQO1, HO-1 and GCLC include resveratrol and xanthohumol [36,37]. Other antioxidant, curcumin activated glutathione S-transferase P1 (GSTP1) gene expression by activating the expression of the luciferase gene from a reporter construct carrying GSTP1-ARE [38].

The article "Piper betle induces phase I & II genes through Nrf2/ARE signaling pathway in mouse embryonic fibroblasts derived from wild type and Nrf2 knockout cells" was published in 2014. Journal: BMC Complement Altern Med.

The increased expressions of Nrf2, NQO1 and GSTA1 genes in WT cells but not in N0 cells further validated our claim that PB is a Nrf2/ARE inducer. McWalter et al. [39] reported that transcription factor, Nrf2 was activated by broccoli seeds and isothiocyanates, with induction of NQO1, GST and GCLC genes and proteins in Nrf2^+/+^ but not in Nrf2^-/-^ mice. Our results are supported by the finding of Yoon et al. [40] who found that sulforaphane increased NQO1 and HO-1 proteins in human proximal cells. Cho et al., [8] have shown that Nrf2 gene was upregulated at least 2-fold higher in Nrf2^+/+^ mice than in Nrf2^-/-^ mice at basal level and also in hyperoxia-induced mice. The possibility of polyphenols in PB such as chavicol or euginol inducing Nrf2 was also reported by a study of Tsai et al., who showed that phenolic compounds from rosemary and carnosic acid induced transcription of Nrf2, ARE luciferase reporter activity and increased expression of NQO1 gene and protein in rat clone 9 cells [41]. Lycopene metabolite, apo-8’-lycopenal that can be found in rat liver and human plasma after consuming lycopene-containing food, induced nuclear translocation, Nrf2-ARE binding activity, HO-1 and NQO1 genes and proteins expression in human hepatoma cell lines, HepG2 [42]. The isothiocyanate, sulforaphane and the flavonoid, epigenin increased gene expression of phase II detoxifying enzyme such as glutathione S-transferase (GSTA1) and UDP-glucuronosyltransferase (UGT1A1) in human colon adenocarcinoma [43]. L-sulforaphane modulates Nrf2-regulated genes including GSH biosynthesis (GCLC), glutathione S-transfreases (GSTA1, GSTA2, GSTA3, GSTM1) and NQO1 in small intestine of Nrf2^+/+^ and Nrf2^-/-^ mice [16].

Our results showed decreased HO-1 mRNA expression after 24 h treatment with PB while its protein level was found to be increased. This finding is similar to a time-course study by Motterlini et al. [44] who showed that HO-1 mRNA expression in bovine aortic endothelial cells reached a maximum after 6 h treatment with 5 μM curcumin and declined after 24 h treatment.

Contrary to many findings, we noted that SOD1 gene and protein were not expressed in WT but were significantly expressed in N0 cells. Others who found similar results reported that the basal level of some antioxidant enzymes may not be under the influence of Nrf2 gene [45,46]. Kwak et al. [47] found that MnSOD gene was 1.31 fold higher in Nrf2-disrupted mice compared to wild-type mice at constitutive levels, suggesting that Nrf2 is an essential factor to modulate many, but not all, antioxidant and phase 2 enzymes. The disruption of Nrf2 gene in Nrf2^-/-^ may alter the basal and inducible expression of some genes including SOD1.

The article "Piper betle induces phase I & II genes through Nrf2/ARE signaling pathway in mouse embryonic fibroblasts derived from wild type and Nrf2 knockout cells" was published in 2014. Journal: BMC Complement Altern Med.

## Conclusion

In summary, our findings indicate that PB activated Nrf2/ARE pathway by dissociating Nrf2 from Keap1, translocating Nrf2 protein into the nucleus, inducing antioxidant response element (ARE), thereby increasing Nrf2-regulated genes (Nrf2, NQO1 and GSTA1) and proteins such as NQO1 and HO-1.

## Competing interests

The authors declare that they have no competing interests.

## Authors’ contributions

WNWH performed experiments and analyzed data. WZWN and YAMY designed the study. KMY gave the cells and general supervision. SM helps for data interpretation on gene expression. All authors read and approved the final manuscript.

## Pre-publication history

The pre-publication history for this paper can be accessed here:

http://www.biomedcentral.com/1472-6882/14/72/prepub
